The article "CNN-Based Personal Identification System Using Resting State Electroencephalography" was published in 2021. Journal: Comput Intell Neurosci.

# CNN-Based Personal Identification System Using Resting State Electroencephalography

**DOI:** 10.1155/2021/1160454

**Published:** 2021-12-13

**Authors:** Yongdong Fan, Xiaoyu Shi, Qiong Li

**Affiliations:** School of Cyberspace Science, Harbin Institute of Technology, Harbin 150001, China

## Abstract

As a biometric characteristic, electroencephalography (EEG) signals have the advantages of being hard to steal and easy to detect liveness, which attract researchers to study EEG-based personal identification technique. Among different EEG protocols, resting state signals are the most practical option since it is more convenient to operate than the other protocols. In this paper, a personal identification system based on resting state EEG is proposed, in which data augmentation and convolutional neural network are combined. The cross-validation is performed on a public database of 109 subjects. The experimental results show that when only 14 EEG channels and 0.5 seconds data are employed, the average accuracy and average equal error rate of the system can reach 99.32% and 0.18%, respectively. Compared with some existing representative works, the proposed system has the advantages of short acquisition time, low computational complexity, and rapid deployment using market available low-cost EEG sensors, which further advances the implementation of practical EEG-based identification systems.

## 1. Introduction

As society enters digital era, identification has become vital in people's work and life. Traditional identification technologies, such as password and hardware token, may be forgotten, lost, or stolen, resulting in identity leakage or identification failure [1]. Such problems can be avoided by using biometric identification techniques, such as face, fingerprints, and gait, which have been widely studied [2–4]. However, face image is easy to be captured, fingerprint may attach to the surface of many objects unconsciously [5, 6], and gait can be recorded and analysed unknowingly, which may be exploited by malicious attacks. In addition, liveness detection is not easy to achieve for these biometrics. The brain signal represented by electroencephalography (EEG) based biometric technique may solve such problems and has become a prominent personal identification method [7].

EEG is a noninvasive imaging technique that records brain electrical signals generated by neurons. First, EEG acquisition requires special measuring devices and electrodes are placed on the surface of the scalp of subjects. When electrodes fail to touch the skin surface of the brain, the quality of EEG signals degrades rapidly [8], which increases the challenge to steal EEG. Second, the brain is one of the best protected organs in the human body, so brain biometrics are not easy to be damaged by external factors. Third, if subjects died, their brain electrophysiological signals could not be generated anymore, so EEG is one of the main clinical indicators for detecting brain death [9]. Finally, brain biometrics can be elicited by numerous distinct brain systems, which makes it possible to change the stored EEG characteristics using a distinct form of brain activity and response [1]. In conclusion, EEG has the advantages of being difficult to steal and damage, easy to detect liveness, and replaceability. Meanwhile, low-cost EEG sensor systems provide an opportunity to implement practical EEG-based identification systems. Compared with medical-grade sensor systems (e.g., Neuroscan 64-channel system, as illustrated in Figure 1(a)), low-cost sensor systems (e.g., EMOTIV EPOC [10], as illustrated in Figure 1(b)) has a gap in the accuracy [11], but their smaller sizes make them more convenient to wear and more acceptable to users. Besides, low-cost sensor systems help to increase the size of subjects and thus avoid system performance failures caused by a lack of sample diversity [12].

The previously proposed identification schemes based on EEG can be categorized into three groups according to EEG protocols: resting states, cognitive tasks, and tasks with external stimuli [13]. In resting states [14], subjects are instructed to relax completely in a quiet environment, and EEG signals of eyes-open or eyes-closed are recorded. In cognitive tasks, such as motor imagery [15], mental workload [16, 17], and driving fatigue [18], subjects normally need to be trained and are required to complete specific tasks according to external cues while collecting their EEG signals [19]. In the tasks evoked by external stimulation, such as visual evoked potential [20] and acoustic stimuli [21], some additional devices are usually necessary to create and collect the appropriate stimulation. Compared with the other two tasks, resting states basically do not need training for subjects and are user-friendly, which has been favored by researchers.

In the present identification study of resting state EEG, most schemes are based on feature extraction. D. L. Rocca et al. [22] proposed a novel approach that focused on spectral coherence-based connectivity between different brain regions and used a Mahalanobis distance-based classifier to identify 10-second EEG signals in 2014. M. Fraschini et al. [23] proposed a scheme that Phase Lag Index was used to calculate a weighted connectivity matrix; then, the nodal eigenvector centrality was computed, and finally genuine-impostor matching scores were computed to identify 12-second EEG signals in 2015. M. Garau et al. [24] proposed the fusion of the above two by feature-level and matching scores-level approaches in 2016, in which an equal error rate of 1.42% was achieved on 12-second eyes-open EEG signals. J.-H. Kang et al. [25] combined 10 single-channel features (seven spectral and three nonlinear) and 10 multichannel features by conducting network analysis into a set of EEG features, and finally a distance-based classifier for authentication was built in 2018. With the rise of deep learning, T. Schons et al. [26] applied CNN to learn the features of resting state EEG in 2018, in which a sliding window of 12 seconds with a stride of 0.125 seconds was performed. The above scheme has two disadvantages in practical applications. (1) The acquisition time is mostly 10 or 12 seconds, which is too long in real-time identification [27]. (2) Recording 64-channel data relies on medical-grade sensors, which have difficulty in user acceptance and cost compared to low-cost sensors. To solve the above problems, Y. Sun et al. [27] proposed a system based on 1D-Convolutional Long Short-Term Memory Neural Network (1D-Convolutional LSTM) in 2019, which allowed only 16-channel EEG signals and 1-second acquisition time. However, this scheme also has two problems. (1) Introducing LSTM into the network will inevitably increase the computational complexity, which has disadvantages in training time and model loading time [27]. (2) Empirically selected channels cannot match market available low-cost sensors, which is not ideal to implement practical systems.

Recently, data augmentation is increasingly used with EEG, which promises to increase the accuracy and stability of EEG classification [28]. Data augmentation generates new samples by transforming existing samples, including noise addition, sampling, recombination of segmentation, Generative Adversarial Network, and so on. For resting state EEG, the commonly used data augmentation algorithm is sliding window, as depicted in Figure 2(a). Since there are no trigger signals in resting state EEG, the fixed window is normally applied to segment the data along the time boundary to generate training samples, as depicted in Figure 2(b). For example, fixed windows of 12 seconds and 1 second were, respectively, used in literature [23, 27]. The sliding window is a generalization form of the fixed window, which includes two attributes window length and stride, and is also suitable for sample segmentation of resting state EEG. For example, data augmentation based on a sliding window of 12 seconds with a stride of 0.125 seconds was implemented in literature [26]. Compared with the fixed window, the sliding window approach creates more samples. However, the present studies on personal identification have not reported the influence of sliding window on the performance.

For identification applications based on resting state EEG, a personal identification system using the CNN model (referred to below as ICAConvNet) is proposed, which applies a sliding window of 0.5 seconds for data augmentation and is validated on the PhysioNet dataset. Experimental results show that the sliding window is effective. When only 14 channels are used, the average Rank-1 accuracy is 99.32% and the average equal error rate can be as low as 0.18%, the performance of which is close to 64 channels. In summary, the proposed system has the advantages of short acquisition time, low computational complexity, and rapid deployment using market available low-cost sensors.

The rest of this paper is arranged as follows: the detailed research methods of the proposed system are introduced in Section 2, including dataset, preprocessing, data augmentation, network architecture, and experimental setup; the experimental results and discussion are given in Section 3; some conclusions are drawn in Section 4.

## 2. Methodology

### 2.1. Overview

Figure 3 shows the overview of the proposed identification system based on resting state EEG. First, in preparation stage, the resting state EEG data are preprocessed and augmented and then are divided into training and testing sets. Second, in enrollment stage, the training sets are trained by ICAConvNet, and the resting state EEG characteristics of all subjects are learned and stored in the system. Finally, in identification stage, test samples are identified by the trained network model in turn, and predicted identities are output. It is worth mentioning that it requires only 0.5-second resting state EEG to achieve rapid identification after enrollment stage.

### 2.2. Data Preprocessing

In order to preserve the original information and learn EEG features as much as possible, the filtering operations are not performed in data preprocessing.

EEG data are commonly a multichannel time series with several tens or even hundreds of sampling electrodes, which are a two-dimensional matrix data structure. Since the magnitude of EEG signals is usually small, in order to avoid gradient explosion and improve the convergence rate in deep learning, Z-score standardization is performed before neural network training, where the mean *μ* and standard deviation *σ* of all signals are calculated for each subject separately, and then a scaling is executed as indicated in the following equation:

(1) $$\begin{array}{c} {\text{Output}}_{i,j}=\frac{{\text{Input}}_{i,j}-\;\mu }{\sigma }, \end{array}$$

where *i*,  *j*,  *μ*, and *σ* refer to the channel, the position in the time dimension, the mean, and standard deviation of all signals, respectively.

### 2.3. Data Augmentation Based on Sliding Windows

The segmented EEG samples for network input can be viewed as a two-dimensional matrix of Channels × Points. In our work, a sliding window of 0.5 seconds with a stride of 0.25 seconds is adopted, and the data sampling rate is 160 Hz, so Channels and Points are set to 64 and 80, respectively. In the experimental section, the impact of sliding windows using different lengths and various strides on system performance will be discussed. Sample segmentation based on sliding window is provided in Algorithm 1.

### 2.4. Neural Network Architecture

Independent component analysis (ICA) [29, 30] is applicable to the problem of blind source separation and is widely used in the analysis of brain signals. Therefore, the observed EEG signals can be separated by ICA, and each separated signal may provide certain identity features. ICA algorithm is based on the following assumptions: the observed matrix *X* is linearly weighted by the independent component matrix S and the mixed matrix A, as given in (2). The goal of ICA is to obtain a separation matrix *W* according to *X* so that the signal matrix *Y* obtained by *W* acting on *X* is the optimal approximation of the independent component matrix *S*, as expressed in the following equation:

(2) $$\begin{array}{c} X\;=\;AS, \end{array}$$

(3) $$\begin{array}{c} Y\;=\;WX\;=\;WAS, \end{array}$$

Corresponding to EEG, the matrices *X*, *S*, and *A* refer to the multichannel time series of subjects, the signal sources inside the brain, and the relationship matrix between the internal signal sources. Inspired by the above ICA algorithm, the collected multichannel EEG signals can also be separated to obtain the approximate original EEG signals of the internal signal sources, and then convolution is used to learn the biometric characteristics of the approximate internal signal sources for identity identification. The details of neural network architecture called ICAConvNet are as follows.

#### 2.4.1. ICA Stage

A matrix with random initial weights is provided as the separation matrix *W*, which is multiplied by the neural network input (matrix *X*) to obtain the approximate internal signal sources matrix *Y*, as shown in equation (3). Taking *Y* as the input of the subsequent convolution operations, the weights of W are iteratively optimized via backpropagation. The ICA stage may be regarded as a kind of implementation of ICA algorithm using neural network.

#### 2.4.2. Convolution Stage

A typical multilayer convolution neural network, including multiple convolution layers and pooling layers, is expected to extract the biometric characteristics of the signal sources inside the brain and compress the parameter scale. The convergent parameters of convolutional kernels are obtained after several iterations of optimization.

#### 2.4.3. Output Stage

The EEG biometric features learned during the convolution stage are combined and outputted. First, the features are flattened and then selected by multiple fully connected layers. Finally, the recognition results are outputted by Softmax function. In order to improve the generalization performance of the system, the dropout function is added between the fully connected layers.

The idea of combining ICA and neural network has been used in functional magnetic resonance imaging [31], but the ICA stage is generally relatively independent from neural network, and the weight optimization of *W* has nothing to do with network. The proposed system integrates ICA into neural network architecture, and the weight optimization of *W* depends on the back propagation of network.

The network architecture is plotted in Figure 4 and implemented using PyTorch [32]. Hyperparameter tuning is performed on the eyes-open session of PhysioNet dataset by the grid search method, when a sliding window of 0.5 seconds with a stride of 0.25 seconds is adopted. After comprehensive consideration of accuracy, complexity, and training time, the main hyperparameters are finally selected as follows. In the ICA stage, the number of internal signal sources is 64. In the convolution stage, three 2-dimensional convolution layers with ELU activation and three max pool layers are adopted. In the output stage, two fully connected layers are established and the dropout rate is 0.5. The final output normalization function is Softmax. The loss function is cross entropy loss, and the optimizer is Adam with a learning rate of 3*∗*10^−3^. The loss function of neural network is shown in equation (4), where *N* represents the number of samples, *O* represents the number of identity labels, *y*_*ij*_ is a function (if the true label of sample *i* is equal to *j*, take 1; otherwise, take 0), and *p*_*ij*_ represents the prediction probability that the label of sample *i* is *j*. All parameters of neural network are shown in Table 1, where *P*, *C,* and *O* represent the number of sample points, the number of sample channels, and the number of identity labels, respectively:

(4) $$\begin{array}{c} Loss=-\sum_{i}^{N}\sum_{j}^{N}y_{ij}\log\left(p_{ij}\right). \end{array}$$

### 2.5. EEG Dataset and Channel Selection

The EEG signals used to verify the proposed system are obtained from a public database called PhysioNet EEG Motor Movement/Imagery Dataset [33–35]. The dataset is available free of charge and all data were collected using a 64-channel BCI2000 system with a sampling rate of 160 Hz. 109 subjects performed 14 different sessions, consisting of two resting baseline sessions and three groups of four motor or motor imagery tasks (T1-T4). Two resting state sessions are chosen, one for 1 minute with eyes-open (EO) and one for 1 minute with eyes-closed (EC).

In recent years, low-cost EEG sensors have made great progress [11], which further increases the possibility that EEG-based identification systems will be used in practical applications. In order to evaluate whether the proposed system works well on these commercial EEG sensors, a series of experiments are conducted using 14, 32, and 64 channels, respectively. The selected 14-channel and 32-channel are based on the EMOTIV EPOC *X* 14 Channel Mobile Brainwear® [10] and EMOTIV EPOC Flex EEG Brainwear® system [36]. Note that the 14 channels of EMOTIV EPOC *X* (AF3, F7, F3, FC5, T7, P7, O1, O2, P8, T8, FC6, F4, F8, and AF4) are all contained in the original 64 channels of PhysioNet dataset. Because the 32 channels of EMOTIV EPOC Flex do not correspond precisely to the original 64 channels, four channels have been reselected (i.e., FT7, TP7, TP8, and FT8). The selected channels in experiments are highlighted in red in Figure 5.

### 2.6. Experimental Setup

To test whether the proposed system can meet the requirements of identification, two experiments were performed on PhysioNet datasets.

#### 2.6.1. Data Augmentation Experiment

The first experiment validates the importance of data augmentation on the system performance. The segmented samples generated by sliding windows with different lengths and strides are trained and tested in turn. The data of the first experiment are all from the eyes-open session, in which the first 48s are divided as the training set and the last 12s as the testing set.

#### 2.6.2. Channel Selection Experiment

The second experiment examines the effects of 14, 32, and 64 channels on the system performance using 5-fold cross-validation. In this experiment, eyes-open session, eyes-closed session, and the union of two resting state sessions are checked in turn.

It should be noted that in both experiments, a sliding window is executed after the training set and testing set are divided. After 1000 training epochs, the experimental results generally tend to be stable, so the termination condition is set as 2000 epochs. The batch size of the training sets is 64. The system performance is evaluated using Rank-1 accuracy, false rejection rate (FRR), false acceptance rate (FAR), and equal error rate (EER). Rank-1 accuracy is used to evaluate the performance in identification scenarios, which is the probability of correctly identifying a user's identity. FRR, FAR, and EER are used to evaluate the performance in authentication scenarios, where the system determines whether a user matches his or her claimed identity [27].

## 3. Results and Discussion

### 3.1. Experimental Results

In the data augmentation experiment, the performance of system using different sliding windows is shown in Table 2. A sliding ratio of 0.5 means that the overlap rate of window is 50%, and a sliding ratio of 1 means that a fixed window is used. When fixed windows were applied, the Rank-1 accuracy of 0.25 seconds, 0.5 seconds, 1 second, and 2 seconds was 99.39%, 98.89%, 94.80%, and 60.86%, respectively. When sliding windows with an overlap rate of 50% were used, the corresponding Rank-1 accuracy was 99.40%, 99.51%, 99.04%, and 92.74%, respectively, and the equal error rates were also improved to 0.15%, 0.06%, 0.19%, and 1.67%. The results show that sliding windows achieved a better performance than fixed windows. Interestingly, the performance of a sliding window of 1 second with a stride of 0.5 seconds was like that of a fixed window of 0.5 seconds, which may be because the number of samples eventually generated by these two segmentation schemes was almost the same. Test accuracy and training loss curves of different windows are plotted in Figure 6. After 2000 rounds of training, the first three augmentation schemes were all in the first echelon and Rank-1 accuracy can reach over 99%, which indicated that the scheme using a window of 0.5 seconds with a stride of 0.25 seconds can achieve excellent performance with less training time.  Figure 7 shows the detection error trade-off (DET) curves of the data augmentation experiment, that is, the relationship between FAR, FRR, and EER, were represented by threshold changes. The smaller EER meant a better performance in authentication scenarios. The scheme using a window of 0.5 seconds with a stride of 0.25 seconds also achieved the best EER of 0.06%. To some extent, for ICAConvNet-based identification system, more samples may bring certain performance gains. In addition, sliding windows with the same window length helped to reduce the acquisition time of the enrollment stage. In summary, a sliding window of 0.5 seconds with a stride of 0.25 seconds is suitable for the proposed system. If the window length is further reduced to 0.25 seconds, the performance is not improved, and the training time is significantly increased.

In the channel selection experiment, referring to comparison results of data augmentation experiment, a sliding window of 0.5 seconds with a stride of 0.25 seconds was used. The performance of 14, 32, and 64 EEG channels in different sessions is shown in Table 3. The selected 14 channels and 32 channels are based on market available EMOTIV EPOC *X* and EMOTIV EPOC Flex, as plotted in Figure 5. According to the experimental results, the performance of 64 channels was generally the best, followed by 32 channels and 14 channels slightly worse. However, although the number of channels was as low as half or even less than a quarter, the performance of the system did not suffer a significant degradation. Therefore, the proposed system had an excellent identification performance even with very few EEG electrodes and can be used to build a practical identification system using low-cost EEG sensors. In addition, the average Rank-1 accuracy can achieve more than 99% in the cross-validation of different sessions, which indicated that the proposed system was effective and robust.

### 3.2. Comparison with Related Works

Our work was compared with the performance of other EEG-based identification systems using PhysioNet dataset, as shown in Table 4. It should be noted that the results selected were from the 14 channels of the union session in the channel selection experiment. The specific result of 5-fold cross verification was that Rank-1 accuracy was 98.152216%, 99.573588%, 99.599431%, 99.819098%, and 99.457294% and EER were 0.465176%, 0.155298%, 0.077230%, 0.064428%, and 0.144111%. The schemes proposed by M. Fraschini et al. [23], M. Garau et al. [24], and T. Schons et al. [26] require 64 EEG channels and 12-second signal segments, which may mean a long wait during the enrollment and identification stages for users. A similar situation exists in the approaches proposed by D. L. Rocca et al. [22] and J.-H. Kang et al. [25]. In the work of S. Yang et al. [37], the accuracy of 99% is achieved on T1-T4 tasks with 9-channel data; however, the window time is increased to 30 seconds. In the 16-channel system proposed by Y. Sun et al., only 1 second of EEG is needed to complete the work, but introducing LSTM into network architecture will inevitably increase the computational complexity, thus increasing the training time required for high identification performance [27], as shown in Table 5. In contrast, the proposed system adopts a sliding window of 0.5 seconds and selects 14 EEG channels based on the existing low-cost EEG sensors, which still has certain advantages in Rank-1 accuracy and EER. Meanwhile, ICAConvNet has a shorter loading time and a faster computing speed, when the testing PC is equipped with an Intel 10700 CPU, a Nvidia 2080Ti GPU, and a Seagate 1 TB HDD. Theoretically, the proposed system has better practicability. Through a combination of ICAConvNet and optimized sliding window, our work has a better overall performance.

## 4. Conclusions

In this paper, a personal identification system using resting state EEG is proposed, which is designed by combining ICA and convolution computation. The number of channels in the system can be as few as 14, and a sliding window of 0.5 seconds is applied for data augmentation. Different sliding window schemes were compared on publicly accessible PhysioNet database to select the optimal data augmentation parameters. In the cross-validation of 109 subjects, Rank-1 of 99.32 ± 0.60% and EER of 0.18 ± 0.15% were achieved, respectively. Compared with related work, our system has certain advantages in the accuracy, computational complexity, and stability, which further advances the implementation of practical EEG-based identification systems.

The identification application of resting state EEG is discussed in this paper. In the future, the characteristics of nonresting state EEG can be further studied. In addition, the challenges faced by EEG-based identification systems in practical application are also worth exploring, such as the permanence and stability of EEG.

## Figures and Tables

**Figure 1:** Typical medical-grade EEG sensor and low-cost EEG sensor. (a) Typical medical-grade sensor, Neuroscan 64-channel Quick cap and (b) typical low-cost sensor, EMOTIV EPOC.

**Figure 2:** The sliding window and the fixed window. (a) The sliding window and (b) the fixed window.

**Figure 3:** Overview of the proposed personal identification system.

**Figure 4:** Neural network architecture.

**Figure 5:** Electrode positions on scalp and their corresponding channels (red represents selected channels, and white represents unused channels). (a) 14 channels, (b) 32 channels, and (c) 64 channels.

**Figure 6:** Test accuracy and training loss curves for different sliding windows. (a) Testing accuracy and (b) training loss.

**Figure 7:** DET curves for different sliding windows.

**Algorithm 1:** Sample segmentation based on sliding windows.

**Table 1:** Neural network parameters.

Layer	Output shape	Description
Input	(None, 1, P, C)	—
ICA	(None, 1, P, 64)	Linear, in_channels: C, out_channels:64
Conv_1	(None, 32, P/2, 64)	Conv2d, in_channels: 1, out_channels:32, kernel: 5 × 3, stride: (2, 1), padding: (2, 1), activation: ELU
Pool_1	(None, 32, P/4, 64)	MaxPool2d, kernel: 2 × 1, stride: (2, 1)
Conv_2	(None, 32, P/4, 64)	Conv2d, in_channels: 32, out_channels: 32, kernel: 3 × 3, stride: (1, 1), padding: (1, 1), activation: ELU
Pool_2	(None, 32, P/4, 32)	MaxPool2d, kernel: 1 × 2, stride: (1, 2)
Conv_3	(None, 32, P/4, 32)	Conv2d, in_channels: 32, out_channels: 32, kernel: 3 × 3, stride: (1, 1), padding: (1, 1), activation: ELU
Pool_3	(None, 32, P/8, 32)	MaxPool2d, kernel: 2 × 1, stride: (2, 1)
Flatten	(None, 32×P/8×32)	Flatten
FC_1	(None, 512)	Linear, in_channels: 32×P/8×32, out_channels: 512
Dropout	(None, 512)	Dropout, p: 0.5
FC_2	(None, O)	Linear, in_channels: 512, out_channels: O
Softmax	(None, O)	log_softmax

**Table 2:** Comparison of the performance of the proposed personal identification systems with different sliding windows.

Window (s)	Sliding ratio	Scale of training set	Training time (min)	Rank-1 (%)	FRR (%)	FAR (%)	EER (%)
0.25	0.5	41747	560	99.40	0.15	0.15	0.15
	1	20928	309	99.39	0.17	0.17	0.17

0.5	0.5	20819	273	**99.51**	**0.06**	**0.07**	**0.06**
	1	10464	136	98.89	0.19	0.19	0.19

1	0.5	10355	147	99.04	0.20	0.18	0.19
	1	5232	74	94.80	1.38	1.38	1.38

2	0.5	5123	85	92.74	1.67	1.68	1.67
	1	2616	43	60.86	10.55	10.55	10.55

Bold values indicate the best performance.

**Table 3:** Comparison of the performance of the proposed personal identification systems with 14-, 32-, and 64-channel EEG signals (positions of the electrodes are shown in Figure 5).

Session	Channels	Rank-1 (%)	FRR (%)	FAR (%)	EER (%)
EO	14	99.04 ± 0.95	0.25 ± 0.21	0.25 ± 0.21	0.25 ± 0.21
	32	99.29 ± 0.81	0.19 ± 0.16	0.19 ± 0.16	0.19 ± 0.16
	64	99.29 ± 0.85	0.21 ± 0.22	0.21 ± 0.22	0.21 ± 0.22

EC	14	99.11 ± 0.85	0.18 ± 0.15	0.19 ± 0.16	0.19 ± 0.15
	32	99.31 ± 0.90	0.15 ± 0.23	0.17 ± 0.24	0.16 ± 0.23
	64	99.44 ± 0.75	0.16 ± 0.19	0.16 ± 0.19	0.16 ± 0.19

EO&EC	14	99.32 ± 0.60	0.18 ± 0.15	0.18 ± 0.15	0.18 ± 0.15
	32	99.64 ± 0.35	0.09 ± 0.06	0.09 ± 0.06	0.09 ± 0.06
	64	99.78 ± 0.23	0.06 ± 0.08	0.07 ± 0.08	0.07 ± 0.08

**Table 4:** Comparison with other EEG-based identification systems using PhysioNet dataset.

Reports	Approach	Session	Subjects	Channels	Sampling rate (Hz)	Window length (s)	Stride (s)	Rank-1 (%)	EER (%)
[22]	PSD and spectral coherence	EO and EC	108	56	160	10	—	100	—
[23]	Eigenvector	EO and EC	109	64	160	12	—	96.90	4.40
[24]	Eigenvector	EO and EC	109	64	160	12	—	—	1.42
[37]	Wavelet coefficients	T1-T4	108	9	160	30	15	99.00	4.50
[26]	CNN	EO and EC	109	64	160	12	0.125	—	0.19
[25]	Eigenvector	EO and EC	109	56	—	12	—	98.93	0.73
[27]	1D-Conv. LSTM	EO and EC, T1-T4	109	16	160	1	—	99.58	0.41
Proposed	CNN	EO and EC	109	**14**	160	**0.5**	**0.25**	99.32 ± 0.60	0.18 ± 0.15

The key parameters used in the proposed system are highlighted in bold.

**Table 5:** Model loading time (T_model_) and averaged execution time for batch testing (T_batch_) for 1D-Convolutional LSTM and the proposed approach.

Model	Channels	T_model_ (s)	T_batch_ (s)
1D-Convolutional LSTM [27] (TensorFlow)	16	17.852	0.065
	32	17.965	0.065
	64	18.477	0.071

Proposed (PyTorch)	14	1.106	0.002
	32	1.102	0.002
	64	1.125	0.002

## Data Availability

PhysioNet EEG Motor Movement/Imagery Dataset can be visited at https://physionet.org/content/eegmmidb/1.0.0/. The code of the proposed system is publicly available at https://github.com/hitfyd/Personal-Identification-System-using-Resting-State-EEG.
